The article "Unlocking faba bean (Vicia fabaL.) potential: How cattle manure and fertilizer boost yields in Kaffa Zone, South-Western Ethiopia" was published in 2025. Journal: Heliyon.

# Unlocking faba bean (*Vicia faba***L**.) potential: How cattle manure and fertilizer boost yields in Kaffa Zone, South-Western Ethiopia

**DOI:** 10.1016/j.heliyon.2025.e41771

**Published:** 2025-01-08

**Authors:** Isreal Zewide, Asrat Ademe

**Affiliations:** a Department of Horticulture, College of Agriculture and Natural Resources, Mizan-Tepi University, Ethiopia; b Department of Plant Sciense, College of Agriculture and Natural Resources, Bonga University, Ethiopia

**Keywords:** Alargeta Kebele, Boka Kebele, Cattle manure, Inorganic fertilizer, *Vicia faba*

## Abstract

This study aimed to optimize faba bean (*Vicia faba***L**.) productivity in Adiyo, southwest Ethiopia, by evaluating the influence of cattle manure (CAM) and blended nitrogen phosphrous sulfur and boron (NPSB) fertilizer rates during the 2023 crop season. Faba bean, a crucial grain legume in Ethiopia, was grown in Alargeta and Boka locations of Adiyo Woreda, Kaffa Zone, and Southwestern Ethiopia. The experiment comprised factorial combinations of four cattle manure (CAM) levels (control., 2.5, 5, 7.5 ha^-1^) and four NPSB fertilizer levels (control., 50, 100, 150 kg ha^−1^) arranged in a Randomized Complete Block Design (RCBD) with three replications. Statistical analysis revealed highly significant combined effects of cattle manure (CAM) and blended nitrogen phosphrous sulfur and boron (NPSB) fertilizer on faba bean harvest index at Alargeta, while Boka exhibited no significance. The highest harvest index (52.5 % and 49.8 %) resulted from cattle manure (CAM) 5 t ha^−1^ + 150 kg ha^−1^ nitrogen phosphrous sulfur and boron (NPSB) fertilizer, equivalent to cattle manure (CAM) 7.5 t ha^−1^ + 150 kg ha^−1^ NPSB at Boka. Conversely, the lowest values (42.8 % and 41.9 %) were observed in control treatments at Alargeta and Boka. cattle manure (CAM) 5 t ha^−1^ + nitrogen phosphorus sulfur and boron (NPSB) 150 kg ha^−1^ exhibited superiority in various parameters, such as the number of branches, plant height, grain yield, hundred seed weight, pods per plant, pod length, and seeds per pod at both locations. This treatment yielded favorable Marginal Rates of Returns (MRRs) of 2595.1 % and 1545.3 %, surpassing the acceptable minimum of 100 %, while control treatments yielded lower net benefits (132,280 and 121,430 ETB ha^−1^). In conclusion, the integrated application of cattle manure (CAM) 5 t ha^−1^ with 150 kg ha^−1^ nitrogen phosphorous sulfur and boron (NPSB) emerged as an economically viable strategy for enhancing faba bean productivity in the study areas, suggesting its potential applicability in similar agro-ecological settings.

## 1 Introduction

The faba bean (*Vicia faba* **L**.), an essential member of the Fabaceae family, has origins in Central Asia, the Mediterranean, and South America, with its primary centers of diversity in North Africa and Southwest Asia [1,2]. Secondary centers are proposed in Ethiopia and Afghanistan. Globally, the faba bean ranks as the third most significant legume, yielding an average annual production of 4.5 million tons [3] The Asia-Pacific region leads global production, contributing 2.7 million metric tons (35.3 %) in 2021 [4].

This cool-season legume plays a critical role in human and livestock diets due to its high protein content and adaptability to diverse agroecological conditions. Known as broad beans, faba beans rank fifth among pulse crops in global production [3]. However, production is often constrained by climatic, edaphic, biotic factors (e.g., diseases, pests, and weeds), and suboptimal agronomic practices.

Ethiopia is the second-largest producer of faba beans worldwide, surpassed only by China. Cultivation spans regions such as Shewa, Arsi, Gojam, Gonder, and Welo, where the crop is a cornerstone of agriculture, supporting food security and soil fertility [3]. Faba beans are vital for human nutrition, fodder production, and environmental sustainability. In 2022, approximately 511,918 ha were devoted to faba bean farming, engaging 3.7 million smallholder farmers [[5], [6]]. Despite this, national yields average only 2.11 tons per hectare, significantly below the global average of 3.7 tons per hectare [4]. Research-managed trials, however, indicate yields of up to 3.5 tons per hectare, emphasizing the potential to close the yield gap through improved practices [7].

Faba bean productivity in Ethiopia is hindered by poor soil fertility, pests, diseases, suboptimal nutrient management, and limited access to high-yielding varieties [8]. Additionally, soil acidity and associated nutrient deficiencies, including nitrogen, phosphorus, potassium, and trace elements, severely limit yields [9].

The Kaffa Zone, a key faba bean cultivation region, faces significant production constraints. Poor soil fertility, high acidity, inappropriate plant densities, and weed infestations are prominent challenges [10],. Soil erosion and leaching in the highlands exacerbate nutrient deficiencies, while limited adoption of improved technologies further suppresses productivity [11]. Average yields in the zone remain below the potential range of 2.3–3.9 tons per hectare.

Integrated nutrient management (INM), which combines organic amendments like cattle manure with inorganic fertilizers such as NPSB (18.9 % N, 37.7 % P_2_O_5_, 6.95 % S, and 0.1 % B), offers a promising strategy to address soil fertility challenges. This approach leverages the strengths of both organic and inorganic fertilizers to enhance soil health, crop growth, and nutrient availability while reducing reliance on expensive synthetic inputs [12,13]. Studies have demonstrated significant yield improvements with INM compared to singular approaches, depending on factors like soil type, climate, and management practices [14,15].

This study investigates the combined application of cattle manure and NPSB fertilizer to optimize faba bean yields in the Kaffa Zone. By identifying optimal application rates and evaluating economic feasibility, the research aims to enhance productivity, promote sustainable farming practices, and improve food security for local farmers.

## 2 Materials and methods

### 2.1 Description of the study area

The experiment took place at two sites within the Adiyo district of the Kaffa zone, Ethiopia [Fig. 1], during the 2023 main cropping season. Alargexa Kebele and Boka Kebele, known for their legume production potential, were chosen for their proximity to Bonga town (19 and 24 km, respectively) and suitable soil conditions. Both areas have Nitosols (red basaltic soils) with a moderately acidic pH around 6.6–6.7, ideal for faba bean growth [16]. While primarily known for cereals and root crops, these areas also dedicate significant land to faba beans (19.7 % of cultivated land).

**Fig. 1:** The study area map of Boka and Alargeta Kebeles, Adiyo district, Kaffa zone South west Ethiopia.

Climate: data.

Both sites have comparable climate characteristics. The patterns of rainfall for a region were characterized by a monomodal distribution with a mostly rainy season of rainfall in the alregata and boka regions. Total rainfall was estimated to be 181.2 mm in Alregata and 213.31 mm in Boka Kebele. The maximum temperatures in alregata varied from 24.39 °C (August) to 24.84 °C (May) and 15.13 °C (August)–19.25 °C (July) in Boka, respectively. Minimum temperature values vary between 20.84 °C (August) and 23.89 °C (May) in Alregata and 16.26 °C (August) to 17.68 °C (May) in Boka, with a minimum value of temperature between 17.29 °C and 16.21 °C in Alregata and Boka locations, respectively. and suited for faba bean requirements(Fig. 2)The weather data comes from the (Wushwush tea plantation meteorological station., 2023)

**Fig. 2:** Monthly rainfall and mean maximum and minimum temperature of Alergta and Boka region in year faba bean growing season

### 2.2 Experimental material

A faba bean named Gebalcho which was released in 2006 was used as a test crop [17].

### 2.3 Cattle manure and soil sampling and analysis

Cattle manure was collected from a local composted farm and collected in sub-samples from a depth of 30 cm (12 inches) towards the center of the pile. Collect more than 10 sub-samples from different areas and depths using a shovel, ensuring full depth of accumulation. and had been recently collected, aged for 3 months The manure was semi-solid. The manure was analyzed for its nutrient content, including pH organic carbon, organic matter, total nitrogen, total phosphorus, a balanced C:N ratio, and a substantial cation exchange capacity. The worker collected semi-solid samples from the spreader either before or during application. For liquid manure, mix the sub-samples in a clean plastic bucket and collect a composite sample. Place the composite sample in a double-bagged 4-L.

Before planting, randomly collect soil samples in a zigzag pattern from 0 to 20 cm depth from multiple locations. Analyze the composite sample at the Jimma Agricultural Research Soil and Plant Analysis Center for the following selected chemical and physical properties: soil pH, cation exchange capacity (CEC), organic carbon, available phosphorus, total nitrogen, available sulfur, and available boron. Ensure uniform slices and volumes of soil in each sub-sample using a vertical auger. Air-dry the samples, grind them with a pestle and mortar, and pass them through a 2 mm sieve. Analyze the composite soil sample for the aforementioned properties using standard laboratory procedures. Soil pH is measured in a 1:2.5 soil-water suspension using a digital pH meter. CEC is determined using the ethanol 95 % extraction method [18].

### 2.4 Treatments and experimental design

To investigate the effect of different cattle manure and NPSB levels: By varying the doses, they were able to see how different nutrient levels affect faba bean growth and yield. The experiment used a randomized complete block design (RCBD) with three replications to examine four rates of blended fertilizer (control, 50, 100, and 150 kg ha^−1^) with four rates of cattle manure (control, 2.5, 5, and 7.5 t ha ^−1^). The treatments were arranged in a factorial design, meaning each NPSB rate was coupled with each manure rate. Cattle dung was spread evenly across the area and absorbed into the soil 30 days before seeding faba bean seeds. Meanwhile, NPSB fertilizer was administered directly while planting. Physico-chemical properties of soil and cattle manure on the experimental sites By strategically selecting locations that encompass a range of representative environmental conditions, including diverse soil types, altitudes, and rainfall patterns, we obtain a more robust and relevant assessment of the treatments' impact on faba bean growth under typical, varied agricultural settings.

#### 2.4.1 Initial physico-chemical properties of soil

The soil analysis conducted in the study area underscores its overall low fertility and slightly acidic nature, as indicated in Table 1. The availability of essential nutrients for crop growth was found to be deficient, likely a consequence of continuous cropping without adequate nutrient replenishment. This practice has led to nutrient depletion and a consequent decline in soil fertility, as reported by Ref. [19] It's worth noting that soil texture, a crucial physical characteristic, determines water intake rate, water-holding capacity, ease of tillage, aeration, and also significantly influences soil fertility [20].

**Table 1:** Soil physico-chemical properties and cattle manure content.

Soil characters	Unit	Value				References	Cattle manure property	Unit	Value
		Alargexa	Rating	Boka	Rating		pH 1:2.5 (H_2_O)		6.93
Texture							Carbon	%	6.8
Sand	%	41		43			%	9.74	
Clay	%	31		30			Total nitrogen	%	0.5
Silt	%	28		27			Total phosphorus	%	0.88
Textural Class	%		clay loam		clay loam	[21]	C:N ratio	–	7.52
Acidity(pH)		6.23	moderately acidic	6.56	slightly acidic	[21]	Cation exchange capacity	cmolc kg^−1^	26.42
Organic carbon	%	1.04	Medium	1.12	medium	[21]			
Total Nitrogen	%	0.17	Moderate	0.18	moderate	[21]			
Available phosphrous	mg kg^−1^	2.4	Very low	2.2	Very low	[21]			
CEC	cmol kg^−1^	23.65	medium	20.94	medium	[21]			
Sulfur	mg kg^−1^	19.2	Deficient	18	Low	[21]			
Boron	mg kg^−1^	0.4	Low	0.6	Low	[21]			

The soil texture analysis results for both Alargeta and Boka sites revealed a dominance of clay, with particle size distributions of 41 % sand, 31 % silt, and 28 % clay for Alargeta, and 43 % sand, 30 % silt, and 27 % clay, classified as clay loam (Table 1). Clay loam soil is categorized as medium-textured, making it particularly well-suited for faba bean production [22]. [23] suggested that the high clay content observed could be attributed to intense weathering caused by prolonged exposure to weathering agents, such as warm temperatures and heavy rainfall, leading to the formation of aluminum and iron oxides. To address the limitations associated with these soil minerals, the addition of sufficient organic matter resources may enhance nutrient retention and availability, supporting sustainable crop production.

The pH values recorded were 6.23 for Alargeta and 6.56 for Boka (Table 1), indicating a moderately acidic soil reaction according to Ref. [24] classification. Climatic factors, such as prolonged rainfall, may contribute to leaching of basic cations from the soil surface and an increment in soil acidity in the study area. The pH values, falling within the slightly acidic range, are considered conducive for faba bean production [25]. The laboratory analysis results for available phosphorus were 2.4 and 2.2 mg kg-1 for Alargeta and Boka, respectively (Table 1). These values classify the soils as very low in available phosphorus content, unsatisfactory for optimal faba bean growth and yield. The low availability of phosphorus could be attributed to fixation in the acidic soils with aluminum (Al) and iron (Fe) oxides, emphasizing the importance of applying phosphorus fertilizer from external sources based on recommended rates.

In terms of total nitrogen content, classified by Ref. [25], the soil samples from both Alargeta and Boka were found to have poor levels of total nitrogen (0.17 % and 0.18 %, respectively, Table 1). This signifies that total nitrogen is a limiting factor for optimum crop growth and yields, potentially due to the unbalanced application of nitrogen-containing fertilizer and continuous cultivation land, leading to a reduction in soil organic matter contents and total nitrogen. Consequently, the application of nitrogen-containing fertilizers is essential to supplement the nitrogen requirement of the crops.

The available sulfur content in the experimental soil was measured at 19.2 and 18 mg kg^−1^ for Alargeta and Boka, respectively (Table 1). According to Ref. [26] guidelines, these values classify the sulfur content as deficient, indicating a need for sulfur-containing fertilizer application to improve soil fertility, crop growth, and yield. The deficiency may be attributed to crop uptake and continuous application of inorganic fertilizers lacking sulfur.

Hot water available boron, considered available to plants, was measured at 0.4 and 0.6 mg kg^−1^ for Alargeta and Boka, respectively (Table 1). According to the rating by Ref. [25], the available boron content of the soil in the experimental sites was low, indicating a deficiency. This may result from crop uptake, leaching, and continuous application of fertilizers lacking boron. Considering that the boron content falls below the critical value recommended for Ethiopian soils, application of boron-containing fertilizers is necessary to optimize soil productivity.

The analysis of soil organic carbon contents for Alargeta and Boka revealed values of 1.04 % and 1.12 %, respectively (Table 1). According to the classification by Ref. [27], these values categorize the organic carbon contents as medium. The medium organic carbon contents of the surface soil may be attributed to organic matter addition through crop residue decomposition on the field.

The cation exchange capacity (CEC) of the experimental soils was measured at 23.65 and 20.94 cmol(+) kg^−1^ for Alargeta and Boka, respectively (Table 1). According to Ref. [18] these values place the soils under the medium range. The medium CEC may be influenced by the high clay content of the soil, as the soil texture of the experimental sites is dominated by clay (Table 1).

#### 2.4.2 Evaluation of the chemical quality of cattle manure

Organic fertilizers, such as farmyard manure (FYM), play a crucial role in enhancing soil fertility by serving as a resilient source of various nutrients. In the conducted laboratory analysis, the FYM used in this experiment exhibited high-quality characteristics, boasting elevated levels of pH (6.93), organic carbon (OC, 6.8 %), organic matter (OM, 9.74 %), total nitrogen (N, 0.5 %), total phosphorus (P, 0.88 %), a balanced C: N ratio (13.6), and a substantial cation exchange capacity (CEC, 26.42 cmolc kg^−1^), as outlined in Table 1.

The FYM employed in the experiment, being slightly alkaline, was applied to improve soil fertility and enhance crop yields. This aligns with findings by Ref. [28], who identified an optimal pH range for various FYM types used in amending soil fertility to boost crop production. According to Ref. [29], a C: N ratio below 10 suggests rapid decomposition. In contrast, a high C: N ratio exceeding 20 may result in nitrogen immobilization as organic matter decomposes, thereby decreasing the availability of nitrogen for crops.

The C: N ratio of the cattle manure used in this study is presented in Table 1, indicating a favorable range for decomposition and subsequent nitrogen availability for crops. As highlighted by Ref. [30] the influence of organic fertilizers extends to their impact on nutrient availability, mineralization and immobilization patterns, their role as an energy source for microbial activities, their contribution as precursors to soil organic matter (SOM), and their ability to reduce phosphorus sorption in the soil.

#### 2.4.3 Experimental procedure and management

Between mid-May and mid-July 2023, the field was cleared, plowed 2–3 times at 15-day intervals using a traditional "Marsha" plow, and leveled manually. Three blocks with 48 plots each were assigned randomly. Well-aged cow dung was sourced from farmers' yards and applied a month before planting at the recommended dose (thoroughly mixed into the 0–20 cm soil layer). NPSB fertilizer was applied at planting (5–8 cm depth). Seeds were planted at the recommended spacing and depth. Standard cultural practices (weeding, fencing, hoeing, maintenance) were followed.

### 2.5 Data collection and analysis

Data were collected on seedling emergence (days), flowering (days), maturity, plant count, nodules per plant, branches per plant, plant height, pods per plant, pod length, seeds per pod, 100-seed weight, grain yield, aboveground biomass, and harvest index. We conducted a normality test and After establishing that the error variances were homogeneous or heterogeneous, a combined or separate analysis of variances was done. Analysis of Variance (ANOVA) procedure of factorial combination of randomized complete block design (RCBD). by using SAS software [31]. The Least Significant Differences (LSD) test was performed at α = 0.05 level of probability to separate means.

### 2.6 Partial budget analysis

Following CIMMYT's partial budget analysis [32], we assessed the economic viability of cattle manure and NPSB fertilizer application. Variable costs (inputs) and gross returns (grain yield) were compared for each treatment. Variable costs included preparation, transportation, and application of both inputs, fertilizer purchase, and harvesting/threshing/winnowing labor. These costs varied based on treatment yield. For example, cattle manure preparation cost was 1320 ETB ton^−1^, transport 620 ETB ton^−1^, and application 250 ton^−1^. Blended NPSB cost was 42 ETB ton^−1^, with 4.4 ETB ton^−1^ for transport and application. Harvest price of faba beans was the prevailing market rate at Bonga (50 ETB ton^−1^). Net returns (NR) were calculated as gross returns (GR) minus variable costs (VC): NR = GR - VC. Other economic analyses followed [33] formula.

## 3 Result and discussion

### 3.1 Crop phenological and vegetative growth parameters

#### 3.1.1 Days to 50 % flowering

The variance analysis revealed a highly significant influence (p < 0.01) on days to 50 % flowering, influenced by main and interaction effects at Alargeta and Boka. Applying 7.5 t ha^−1^ CAM with 150 kg ha^−1^ blended NPSB fertilizer significantly delayed flowering (57.3 and 49.3 days) at Alargeta and Boka. The latest days to 50 % flowering at Boka aligned with CAM 7.5 t ha^−1^ with 100 kg^−1^ blended NPSB fertilizer, while the earliest results (43.6 and 40.3 days) were noted at Alargeta and Boka with 50 kg ha^−1^ blended NPSB fertilizer and control treatments (Table 2). Low Temperature in Alargeta plays a crucial role in flowering time.or leading to cooler conditions that could delay flowering.The delay in flowering, possibly due to increased levels of nitrogen in NPSB and cattle manure, led to excessive haulm development, as suggested by Ref. [[34], [35]]. This concurs with findings by Ref. [36], who observed delayed flowering and maturity in potatoes with nitrogen, phosphorus, and sulfur fertilizer applications. The delayed flowering could be attributed to the increased application rate of CAM 7.5 t ha^−1^ and 150 kg blended NPSB ha^−1,^ resulting in longer flowering times, while zero and manuring plots required a shorter time. Manure application increased soil pH, reduced aluminum solubility, and promoted plant growth [9]. Delayed flowering contributes directly to higher yields per unit of land and time. This increases food availability, enhances farmer income, and reduces reliance on imported food, boosting food security [[37], [38]]

**Table 2:** The effects of NPSB and Cattle manure on phenological parameters of faba bean over the location.

NPSB kg ha^−1^	CAM t ha^−1^	Alargeta		Boka	
		DF	DPM	DF	DPM
control.	control.	44.0^i^	121.3^h^	40.3^k^	111.0^i^
	2.5	45.3^gh^	123.3^g^	42.0^ji^	113.3^h^
	5	45.3^gh^	125.6^f^	43.0^gih^	115.3^g^
	7.5	49.3^d^	126.6^f^	44.0^gfe^	117.6^e^
50	0	43.6^i^	124.3^g^	41.3^jk^	113.0^h^
	2.5	45.3^gh^	126.3^f^	43.3^gfh^	115.0^g^
	5	48.3^ed^	128.6^e^	45.0d^ec^	116.3^f^
	7.5	51.0^c^	131.0^d^	45.6^c^	118.6^d^
100	0	44.6^ih^	126.3^f^	42.0^ji^	113.6^h^
	2.5	46.3^gf^	131.0^d^	44.3^dfe^	118.0^ed^
	5	49.3^d^	132.0^d^	47.3^b^	119.6^c^
	7.5	51.3^c^	134.3^c^	49.0^a^	122.0^b^
150	0	46.6^f^	128.3^e^	42.6^ih^	115.6^gf^
	2.5	48.0^e^	133.6^c^	43.6^gfh^	116.3^f^
	5	55.0^b^	138.3^b^	45.3^dc^	118.3^ed^
	7.5	57.3^a^	143.6^a^	49.3^a^	124.3^a^
LSD (0.05)		1.91	1.12	1.04	0.98
p value		∗∗	∗∗	∗∗	∗∗
CV(%)		3.4	4.5	2.3	3.6

Where: DF = days to 50 % flowering, DPM = days to 90 % physiological maturity, LSD = list significant difference, CV = coefficient of variance. ∗∗, and ∗ indicate significant differences at 1 % (p ≤ 0.01), and 5 % (p ≤ 0.05 level of significance, respectively; Letters in column 'a', 'b', 'c', etc represents respective mean values from highest to lowest.

#### 3.1.2 Days to 90 % maturity

The analysis demonstrated a highly significant (p < 0.01) influence on days to 90 % maturity, affected by the main and interaction effects of CAM and NPSB application rates in both locations. CAM 7.5 t ha^−1^ with 150 kg ha-1 blended NPSB fertilizer delayed maturity (124.3 and 143.6 days) at Boka and Alargeta, while zero (control) treatments exhibited the shortest duration to maturity (111 and 121.3 days) at Boka and Alargeta this deliances in alrgata might be suitable microenvironment temperature, light, or rainfall) (Table 2). The difference between the earliest and latest days to 90 % maturity (Boka 13.3, Alargeta 22.3 days) was remarkable. The crop matured later, possibly due to the application of CAM 7.5 t ha^−1^ and 150 kg ha^−1^ blended NPSB fertilizer, increasing maturity times, while zero plots matured quickly. The incremental CAM manure and P fertilizer rates extended faba bean maturity at both locations. This difference may stem from nutrient shortages in untreated plots and sufficient nutrient supply in treated plots. Nitrogen availability in NPSB fertilizer and farmyard manure might be the cause of delayed faba bean maturity. Plants receiving high amounts of inorganic and organic fertilizer remained vegetative for a longer time compared to control plots, consistent with findings on potatoe [33]. Physiological maturity was earliest at Boka and latest at Alargeta with the same application of CAM 7.5 t ha^−1^ and 150 kg ha^−1^ blended NPSB fertilizer. This aligns with [39], attributing delayed physiological maturity to increased NPSB and CAM application, enhancing vegetative growth rather than physiological maturity. This result concurs with [40], stating that nitrogen fertilizer significantly affects days to 90 % physiological maturity in black cumin.

Similar to flowering time, longer time to maturity is advantageous. A longer period to reach maturity can:

Faster maturity directly leads to greater yields, which helps improve food availability and farmer income [41].

#### 3.1.3 Number of nodules per plant

The main and interaction effects of manure with blended NPSB fertilizer rate significantly influenced the number of nodules per plant at both locations (p < 0.01). The highest nodules (72.9 and 73.0) were observed with CAM 5 t ha^−1^ and 150 kg ha^−1^ blended NPSB at Alargeta, and CAM 7.5 t ha^−1^ with 150 kg ha^−1^ blended NPSB at Boka. In contrast, the lowest nodules (50.1 and 48.0) were recorded in the control treatment at both experimental areas (Table 3). The increased nodulation with blended NPSB fertilizer application could be attributed to the need for an adequate amount of phosphorus crucial for plant growth, nodule formation, and N_2_ fixation [42]. Other studies, including [43], supported this outcome, suggesting that manure application enhances indigenous rhizobium populations, fostering a conducive environment for bacterial proliferation. The rise in nodule numbers may be linked to improved soil rhizobium conditions due to increased phosphorus and micronutrient content from farmyard manure. Similarly [44,[45], [46]], reported significantly higher nodule numbers with integrated inorganic-organic fertilizer applications for lentils and peanuts, respectively.

**Table 3:** The effects of NPSB and Cattle manure on growth parameters.

NPSB kg ha^−1^	CAM t ha^−1^	Alargeta			Boka		
		NN	NB	PH	NN	NB	PH
control.	control.	50.1^f^	1.6^m^	151.2^n^	48.0^k^	1.0^j^	139.8^n^
	2.5	53.7^fed^	2.0^k^	156.4^l^	53.3^ji^	1.2^i^	145.0^l^
	5	55.4^fecd^	2.3^ji^	160.3^i^	54.3^ji^	1.4^fe^	145.0^l^
	7.5	58.2^ecd^	2.46^g^	164.6^f^	58.0^ghef^	1.6^d^	151.8^f^
**50**	0	52.0^fe^	1.9^l^	153.3^m^	53.0^j^	1.3^hi^	142.5^m^
	2.5	54.3^fed^	2.2^j^	157.5^k^	55.3^jhi^	1.4^fg^	146.1^k^
	5	56.2^fecd^	2.5^fg^	161.8^h^	57.3^ghf^	1.6^d^	150.4^h^
	7.5	59.3^bcd^	2.6^e^	165.3^e^	60.3^de^	1.7^c^	153.9^e^
100	0	55.2^fecd^	2.3^hi^	156.4^l^	56.0^ghi^	1.3^hg^	144.7^l^
	2.5	57.4^ecd^	2.4^hg^	162.2^g^	58.3^gef^	1.4^fe^	150.8^g^
	5	62.2^bc^	2.6^e^	165.7^d^	63.3^c^	1.6^dc^	154.3^d^
	7.5	65.4^b^	2.8^d^	173.2^b^	66.6^b^	1.8^b^	161.8^b^
150	0	58.7^becd^	2.6^fe^	158.9^j^	59.6^def^	1.5^e^	147.5^j^
	2.5	60.3^bcd^	3.3^c^	165.4^e^	61.3^dc^	1.6^d^	154.0^ed^
	5	72.9^a^	3.8^a^	180.3^a^	67.3^b^	2.3^a^	165.9^a^
	7.5	65.8^ba^	3.5^b^	173.2^b^	73.0^a^	1.9^b^	161.8^b^
LSD (0.05)		7.18	0.1141	0.2423	2.81	0.0836	0.3474
p value		∗∗	∗	∗∗	∗∗	∗	∗∗
CV(%)		7.3	5.3	5.2	2.8	3.2	3.1

*NN= Number of nodules* per *plant, NB number of branches* per *plant, PH = plant height, LSD = list significant differences, CV = coefficient of variance*. ∗∗, and ∗ indicate significant differences at 1 % (p ≤ 0.01), and 5 % (p ≤ 0.05 levels of significance, respectively; *Letters in column 'a', 'b', 'c', etc represents respective mean values from highest to lowest*.

Higher nodule numbers contribute directly to increased crop yields without external nitrogen input. This reduces reliance on synthetic fertilizers, which are expensive, environmentally damaging [47].

#### 3.1.4 Number of branches

Significant effects (p < 0.05) of the main and interaction factors of manure and blended NPSB fertilizer application rate on the number of branches per plant were observed at both locations. The highest branches (3.8 and 2.3 cm) resulted from manure 5 t ha^−1^ with 150 kg ha^−1^ NPSB at Alargeta and Boka, while the lowest branches (1.6 and 1) were noted in the control treatment at both locations (Table 3). Overall, the combination of the highest rate of 150 kg NPSB ha^−1^ with 5 t ha^−1^ CM yielded optimal results. This aligns with [48], who found increased branches with combined FYM and P application in faba beans. **[**46] reported similar results with combined applications of N, P, K, S, Zn, and B increasing primary branches per plant [49]. also observed increased pH after organic and inorganic fertilizer applications, leading to enhanced nutrient uptake and increased crop growth. In contrast [9], found that combining P and FYM did not affect the number of branches per plant in chickpeas. Plant height.

Analysis of variance revealed a highly significant (p < 0.01) impact of both main and interaction factors on plant height at both locations. However, at Boka, the interaction effect (p < 0.05) did not significantly influence faba bean plant height. The tallest plants (180.3 and 165.9 cm) were observed at Alargeta and Boka with an application rate of CAM 5 t ha^−1^ with 150 kg ha^−1^, while the shortest plants (151.2 and 139.8 cm) were recorded in the control treatment at Alargeta and Boka locations, respectively (Table 3).

The heightened plant growth in faba beans could be attributed to the CAM application at 5 t kg ha^−1^ with 150 kg ha-1 blended fertilizer, potentially increasing N2 availability, fostering maximum vegetative growth. This aligns with (Shiberu et al., 2023), who noted the highest plant height (49.20 cm) with increased NPSB application and 7.5 t ha^−1^ cattle manure, suggesting enhanced N_2_ uptake during the growth period leading to increased cell size, elongation, and division. Conversely, the control treatment resulted in the lowest height (33.20 cm). The variation in plant height among treatments may be due to the differing manure rates and the impact of higher P_2_O_5_ rates on meristematic cell activities crucial for faba bean's vegetative growth.

This outcome concurs with [50], who reported increased faba bean plant height with rising nitrogen and phosphorus fertilizer. Similarly [51], found significant height enhancement in faba beans with P_2_O_5_ application on acidic Nitosols in Ethiopia [9]. noted increased common bean plant height with rising N2 levels, while [11] found that cattle manure and NPSB significantly increased common bean plant height.

The tallest plants with NPSB application may be due to phosphorus's positive impact on root proliferation, nodulation, and protoplasm synthesis, leading to increased plant height, more rapid dry matter production, and a higher number of branches [22]. Nitrogen and sulfur, involved in chlorophyll formation, likely contributed to vegetative growth and increased plant height [52].

Conversely, the shortest plants in unfertilized plots were a result of the soil's low nutrient-supplying capacity, leading to reduced soil fertility levels [51]. emphasized that nitrogen, as a primary limiting nutrient, plays a vital role in plant growth, contributing to chlorophyll formation, increased photosynthetic activity, vigorous vegetative growth, and taller plants.

Increased branching contributes to higher yield potential, thus directly supporting food security.

### 3.2 Yield components and yield

#### 3.2.1 Number of pods per plant

The analysis of variance underscored the profound significance (p < 0.01) of both main and interaction effects of manure and blended NPSB fertilizer application on the number of pods per plant at both locations. The highest pod count (55.0 and 42.0) occurred at Alargeta and Boka with an application rate of CAM 7.5 t ha^−1^ with 150 kg ha^−1^, statistically comparable to CAM 5 t ha^−1^ with 150 kg ha^−1^ fertilizer rates. In contrast, the lowest pod count (34.5 and 22.1) emerged from the 50 kg ha^−1^ blended fertilizer rate at Alargeta and the control treatment at Boka (Table 3).

The increase in pod numbers could be attributed to the higher CAM rate with a blended NPSB fertilizer. This aligns with [48], who reported an increased number of pods per plant in faba beans with integrated FYM and P. Similarly [53], observed significant pod increases in faba beans with chemical, bio-fertilizer, and organic treatments [49]. attributed the rise in pod count to FYM's role in promoting seed germination, root growth, and improved soil conditions, enhancing nutrient supply and water retention [50]. noted that increased leaf area and dry mass production, influenced by N_2_ and P_2_O_5_ application, can contribute to higher pod production.

this directly reflects the plant's reproductive capacity. A higher number of pods indicates greater potential yield. Factors like plant health, pollination success, and environmental conditions influence this number [51].

#### 3.2.2 Pod length

The analysis of variance indicated that pod length in faba beans was significantly (p < 0.05) influenced by the main factor of blended NPSB fertilization and interaction effect at Alargeta and highly significantly (p < 0.01) influenced by the main factor of CAM and NPSB fertilization, with a significant (p < 0.05) interaction effect at Boka. The longest pods (9.3 and 6.7 cm) resulted from CAM 5 t ha^−1^ with 150 kg ha^−1^ of blended NPSB fertilization at both locations, while the shortest (6.9 and 4.0 cm) pods were observed in the control treatment at both locations (Table 3).

The positive impact of organic manure on growth and yield attributes may be due to the additional nutrient supply and improvements in soil properties [54]. Enhanced vegetative growth and nutrient availability from organic manure may contribute to longer pod lengths [52]. These results align with the findings of [55,56], who reported increased pod length in broad beans with organic manure and chemical fertilizer. **[**54 found that manure and NPK application significantly increased growth and yield parameters, including pod length, in garden peas. Longer pods generally contain more seeds, contributing to higher yield per plant. **[**55**]**.

#### 3.2.3 Number of seeds per pod

The analysis of variance demonstrated a significant (p < 0.05) impact of both manuring and blended NPSB fertilization main factors, along with their interaction effect at both locations, on the number of seeds per pod. The highest mean number of seeds per pod (3.7) resulted from the combined application of CAM 5 t ha^−1^ with 150 kg ha^−1^ blended NPSB at Alargeta, while (2.8) was obtained from the combined application of CAM 7.5 t ha^−1^ with 150 kg ha^−1^ blended NPSB at Boka, statistically on par with the fertilizer rate of CAM 5 t ha^−1^ with 150 kg ha^−1^. The lowest mean number of seeds per pod (2.4 and 1.2) was recorded from the control treatment at Alargeta and Boka, respectively (Table 3).

The observed increase in seed numbers could be attributed to the slow release of nutrients from organic matter, complemented by inorganic fertilizers. This enhances microbial growth, expediting organic manure decomposition, and subsequently increasing nutrient availability. This finding aligns with **[**56**]**, who reported a significant increase in lentil pod numbers with phosphorus fertilization due to its cumulative effect on cell division and balanced nutrition. Adequate N_2_ and P_2_O_5_ availability may have facilitated more primary and secondary branch production and increased plant height, contributing to higher pod production.

Moreover, the increase in pods per plant could be associated with expanded leaf area, as additional N encourages more reproductive nodes. Consistent with these results [57,58], found positive influences of manure and phosphorus fertilizer on the number of pods per plant and seeds per pod in faba beans. Additionally [59], reported that the application of 7.5 t ha^−1^ manure with P_2_O_5_ fertilizer resulted in the highest number of pods per plant and seeds per pod in faba beans.

combined with pod length and number of pods, determines the overall seed production per plant. A higher number of seeds per pod significantly contributes to increased yield [60].

#### 3.2.4 Hundred seed weight

The analysis of variance indicated a highly significant (p < 0.01) influence of both manure and blended NPSB fertilization, including their interaction effect, on the hundred seed weight of faba beans at both locations. The highest hundred seed weights (88.6 and 82.6 g) resulted from the integrated application of 5 t ha^−1^ CAM with 150 kg ha^−1^ blended NPSB fertilization at Alargeta and Boka, respectively. In contrast, the lowest values (62.3 and 56.3 g) were recorded from the control treatment at both locations (Table 4).

**Table 4:** The effects of Cattle Manure and NPSB Yield parameters of faba bean.

NPSB kg ha-^1^	CAM t ha^−1^	Alargeta							Boka						
		NPP	PL	NSP	ADGB	HSW	GRY	HI	NPP	PL	NSP	ADGB	HSW	GRY	HI
control.	control.	34.7^l^	6.9^j^	2.4^i^	6181.0^l^	62.3k	2645.6^l^	42.8^k^	22.1^l^	4.0^g^	1.2^i^	5781.6^p^	56.3^h^	2428.6^k^	41.9^g^
	2.5	35.6^jk^	7.3^h^	2.6^hg^	6345.3^j^	67.6^h^	2861.0^i^	45.1^h^	24.5^k^	4.3^gf^	1.5^h^	6144.0^n^	61.6^f^	2679.0^j^	43.6^f^
	5	37.5^hi^	7.5^g^	2.7^f^	6580.3^e^	72.3^g^	3033.0^g^	46.1^g^	27.9^h^	4.4^f^	1.6^h^	6379.0^j^	66.3^e^	2848.6^hi^	44.6^e^
	7.5	38.8^g^	8.0^e^	2.9^ed^	6856.0^d^	77.3^e^	3041.6^g^	47.2^ef^	29.8^g^	4.8^e^	1.8^g^	6555.0^f^	62.3^f^	2959.6^d^	45.1^f^
50	0	34.5^k^	7.0^i^	2.5^hi^	6204.0^l^	65.0^j^	2695.3^k^	43.4^j^	25.5^j^	4.1^g^	1.5^h^	6103.6^o^	57.6^g^	2702.3^g^	44.2^gh^
	2.5	38.5^hg^	7.4^h^	2.6^g^	6386.3^i^	72.0^g^	3003.0^h^	47.0^f^	32.5^f^	4.9^e^	2.1^e^	6256.6^k^	65.3^e^	2821.0^fg^	45.0^f^
	5	40.1^f^	7.9^e^	2.8^ef^	6557.6^f^	76.0^f^	3108.0^f^	47.4^edf^	32.7^f^	5.7^c^	2.3^d^	6457.6^h^	69.6^d^	2992.6^e^	46.3^cd^
	7.5	43.4^d^	8.3^d^	2.9^d^	6790.6^e^	80.0^c^	3238.0^e^	47.7^ed^	35.0^e^	5.8^c^	2.4^c^	6690.6^d^	74.0^c^	3122.67^c^	46.6^cd^
100	0	34.7^k^	7.4^hg^	2.7^f^	6313.6^k^	65.3^j^	2768.3^j^	43.8^ji^	27.3^i^	4.5^f^	1.9^f^	6213.6^m^	61.3^f^	2862.6^h^	46.0^d^
	2.5	42.0^e^	7.8^f^	2.7^f^	6524.6^g^	76.0^f^	3091.0^f^	47.3^ef^	34.6^e^	5.3^d^	2.16^e^	6424.6^i^	70.0^d^	2975.6^fe^	46.3^cd^
	5	43.9^d^	8.4^d^	2.9^d^	6779.6^e^	80.0^c^	3244.0^e^	47.8^d^	36.5^d^	5.8^c^	2.3^d^	6679.6^e^	74.0^c^	3128.6^c^	46.8^cd^
	7.5	46.9^c^	8.8^b^	3.1^c^	6965.3^c^	84.0^b^	3367.0^d^	48.3^c^	38.2^c^	6.3^b^	2.6^b^	6898.6^b^	78.0^b^	3251.6^b^	47.1^cb^
150	0	36.4^ji^	7.9^f^	2.9^d^	6446.6^h^	66.6^i^	2849.0^i^	44.2^i^	29.4^g^	4.7^e^	2.0^fe^	6246.6^l^	69.0^d^	2889.0^hg^	46.2^cd^
	2.5	46.3^c^	8.5^c^	3.1^c^	6779.6^e^	79.0^d^	3426.3^c^	50.5^b^	38.4^c^	5.6^c^	2.5^c^	6479.6^g^	73.0^c^	3111.0^dc^	48.0^b^
	5	55.06^a^	9.3^a^	3.7^a^	7559.33^a^	88.6^a^	3966.33^a^	52.5^a^	42.0^a^	6.7^a^	2.8^a^	6729.6^c^	82.6^a^	3569.0^a^	49.8^a^
	7.5	53.8^a^	8.9^b^	3.3^b^	6965.33^b^	86.3^b^	3516.72^b^	51.0^b^	40.5^b^	6.3^b^	2.8^a^	7157.6^a^	80.3^ba^	3297.0^b^	49.0^a^
LSD(0.05)		1.6904	0.1091	0.0985	2.6041	31.38	2.6041	0.4364	0.4364	0.4846	0.2398	0.1076	0.3881	2.7632	49.497
p-value		∗∗	∗	∗	∗∗	∗∗	∗∗	∗∗	∗∗	∗∗	∗∗	∗∗	∗∗	∗∗	∗∗
CV(%)		7.4	7.4	8.2	9.6	10.2	9.6	0.98	0.98	5.8	6.7	5.1	6.0	5.0	8.1

*Where; NPP = number of pods* per *plant, PL = pod length, NSP = number of seeds* per *pod AGDB = above-ground dry biomass, HWS = hundred seed weight, GRY = grain yield HI = harvest index LSD = list significant difference, CV = coefficient of variance.* . ∗∗, and ∗ indicate significant difference at 1 % (p ≤ 0.01), and 5 % (p ≤ 0.05 level of significance, respectively; *Letters in column 'a', 'b', 'c', etc represents respective mean values from highest to lowest*.

This notable increase in seed weight can be attributed to the combined application of optimal organic and inorganic fertilizers. The augmented hundred seed weight with increasing NPSB and FYM levels suggests sustained nutrient supply throughout the growth period, mitigating nutrient stress and promoting microbial activity. The strengthened root system further enhances soil exploration, nutrient mobilization, and uptake efficiency. This, in turn, accelerates metabolic processes, leading to improved photosynthesis and efficient translocation of photosynthates, resulting in higher seed weight. This aligns with [61], reporting significantly higher 100 seed weight with the integrated use of NPK and FYM.

This measures the weight of 100 seeds and is an indicator of seed size and quality. Larger seeds generally indicate better germination rates and seedling vigor, contributing to better establishment and ultimately higher yields [62].

Moreover, the higher seed weight can be attributed to the significant contribution of additional N from N2-fixation and FYM to chemical fertilizers, crucial for amino acids and various biological compounds involved in photosynthesis and seed weight enhancement. This result is consistent with [63], who associated increased seed size and 100-grain weight with phosphorus fertilization.

#### 3.2.5 Above-ground dry biomass

The analysis of variance highlighted a highly significant (p < 0.01) influence of manuring and blended NPSB fertilization, along with their interaction, on the total above-ground dry biomass of faba beans at both locations. The highest biomass (7559.3 and 7157.6 kg ha^−1^) resulted from the combined application of 5 t ha^−1^ CAM with 150 kg ha^−1^ blended NPSB fertilizer, while the lowest values (6181.0 and 5781.6 kg ha^−1^) were recorded from the control treatment at Alargeta and Boka, respectively (Table 4).

The enhanced biomass observed with the combined application of blended NPSB fertilizer and farmyard manure may be attributed to increased nutrient availability in the soil. Efficient utilization of nutrients due to improved soil chemical and physical properties, facilitated by farmyard manure, contributes to increased biomass. The study underscores that supplying adequate cattle manure and blended fertilizer to faba beans leads to higher plant biomass during harvesting. the total dry weight of the plant's above-ground parts (stems, leaves, pods). It' showsoverall plant growth and maximum resource utilization [64].

The response in dry biomass could be attributed to the rapid expansion of dark green foliage intercepting and utilizing more light energy for photosynthesis. Increased photosynthate production likely contributed to higher plant height, the number of pods per plant, number of seeds per pod, and the number of branches per plant, ultimately influencing higher seed and straw yields. This finding aligns with the reports of [65], associating increased dry matter yield of chickpeas with phosphorus and sulfur application. Similarly, increased dry biomass yield in response to higher phosphorus application rates can be attributed to improved root growth and leaf expansion, enhancing nutrient exploration.

#### 3.2.6 Grain yield

The analysis of variance revealed a highly significant (p < 0.01) influence of both manuring and blended NPSB fertilizer application on faba bean grain yield at both locations. The highest grain yield (366.3 and 3569.0 kg ha^−1^) resulted from the integrated application of 5 t ha^−1^ CAM with 150 kg ha^−1^ blended NPSB fertilization, while the lowest yield (2645.6 and 2428.6 kg ha^−1^) was recorded from the control treatment at Alargeta and Boka, respectively (Table 4).

The increment in grain yield can be attributed to the simultaneous increases in hundred-grain weight, pod number per plant, and seed number per plant, facilitated by NPS and enhanced phosphorus and nitrogen availability due to manure. This positive response may be due to increased nutrient absorption from NPSB and manure, leading to increased reproductive structure formation and efficient assimilate production for seed filling. This result is in agreement with [66], who reported significant effects of different combinations of manure and N fertilizer treatments on groundnut grain yield and biological yield. Additionally, the interaction effect of organic manures with 150 kg ha^−1^ blended NPSB fertilization significantly increased chickpea grain yield [67].

Improving grain yield is crucial for enhancing food security in Ethiopia, where faba bean is a significant dietary staple. [68], emphasizing that the maximum yield of a legume crop depends on its yield components, such as the number of branches per plant, pods per plant, seeds per pod, and seed weight. Overall, the application of 7.5 t ha^−1^ CAM with 150 kg ha^−1^ blended NPSB fertilizer increased grain yield by 33.1 % and 31.96 % compared to control treatments at both locations. When compared to the national average yield, the application of 7.5 t ha ^−1^ CAM with 150 kg ha^−1^ blended NPSB fertilizer led to a 53.8 % increase in faba bean grain yield. All manuring and sole blended NPSB fertilization produced lower grain yields than the integrated approach.

#### 3.2.7 Harvest index

The harvest index, a vital indicator of nutrient and dry matter allocation efficiency in crops was highly significantly influenced by both manuring and blended NPSB fertilization, including their interaction, at Alargeta and Boka locations (p < 0.01). The highest harvest index values (52.5 and 49.8 %) resulted from applying 5 t ha^−1^ CAM with 150 kg ha^−1^ blended NPSB fertilizer. In comparison, the lowest values (42.8 and 41.9 %) were recorded from the control treatment at Alargeta and Boka, respectively (Table 4).

The increased harvest index with the application of 5 t ha^−1^ 150 kg ha^−1^ blended NPSB fertilizer can be attributed to enhanced photo-assimilate production and efficient partitioning to grains over straw. This result is consistent with the findings of [69], who observed a rising trend in harvest index with phosphorus application. The highest harvest index values at the highest CAM and blended NPSB fertilizer rate may be attributed to their synergistic effect on soil fertility, providing essential nutrients for plant uptake and improved vegetative growth. Similar findings in potatoes by Ref. [9] reported a 15 % and 16 % increase in harvest index due to FYM alone and combined half FYM and blended fertilizer application compared to control.

In summary, the integrated approach of 5 t ha^−1^ CAM with 150 kg ha^−1^ blended NPSB fertilizer demonstrated significant positive effects on hundred seed weight, above-ground dry biomass, grain yield, and harvest index of faba beans. This approach maximizes nutrient availability, enhances vegetative growth, and optimizes photo-assimilate partitioning for increased seed weight and yield. Significant increases in hundred seed weight, above-ground dry biomass, grain yield, and harvest index all result in a higher overall yield of faba beans. This increased yield increases the supply of a critical protein source for Ethiopian populations, helping to improve food security by reducing malnutrition and hunger levels.

### 3.3 Economic analysis

Economic feasibility of fertilizer application in cropping seasons is contingent upon the potential crop response and fertilizer prices [33]. Identifying treatments offering maximum returns to farmers requires marginal rate of return (MRR) analysis on non-dominated treatments, where a 100 % MRR indicates a viable option for farmers [33].

Partial budget analysis of faba bean reveals significant impacts from varying rates of CAM and blended NPSB fertilizer (Table 5, Table 6). Treatment T15, involving 5 t ha^−1^ cattle manure and 150 kg ha^−1^ blended NPSB fertilization, showcased the highest net return (187,775 and 167,010 ETB ha-1), establishing its economic superiority. Increasing the integrated CAM and NPSB blended fertilizer application rates amplified net benefits, indicating improved soil conditions and subsequently enhanced grain yield. Discrepancies in yield between Alargeta and Boka underscored agroecological variations favoring faba bean production in Alargeta.

**Table 5:** A partial budget analysis is needed to estimate the net benefit of the combined use of CM and NPSB for Faba bean production at the Alargeta location.

Alargeta												
Treatment	UUY (kg ha^−1^)	AGY (kg ha^−1)^	GFB (ETB)	VC NPSB(ETB)	VC CAM (ETB)	Transportation cost (ETB)		Application cost ETB		TVC (ETB)	NFB (ETB)	MRR (%)
						NPSB (ETB)	CAM (ETB)	NPSB (ETB)	CAM (ETB)			
T 1	2963.1	2645.6	132280	0	0	0	0	0	0	0	132280	
T 2	3204.3	2861	143050	0	1320	0	620	0	250	2190	140860	ND
T 5	3018.7	2695.3	134765	2140	0	50	0	220	0	2410	132355	D
T 3	3397	3033	151650	0	2640	0	1240	0	500	4380	147270	ND
T 6	3363.4	3003	150150	2140	1320	50	620	220	250	4600	145550	D
T 9	3100.5	2768.3	138415	4280	0	100	0	440	0	4820	133595	D
T 13	3190.9	2849	142450	5350	0	150	0	660	0	6160	136290	D
T 4	3630.6	3041.6	152080	0	3960	0	1860	0	750	6570	145510	D
T 7	3481	3108	155400	2140	2640	50	1240	220	500	6790	148610	ND
T 10	3461.9	3091	154550	4280	1320	100	620	440	250	7010	147540	D
T 14	3837.5	3426.3	171315	5350	1320	150	620	660	250	8350	162965	ND
T 8	3626.6	3238	161900	2140	3960	50	1860	220	750	8980	152920	D
T 11	3633.3	3244	162200	4280	2640	100	1240	440	500	9200	153000	D
T 15	4442.3	3966.3	198315	5350	2640	150	1240	660	500	10540	187775	ND
T 12	3771	3367	168350	4280	3960	100	1860	440	750	11390	156960	D
T 16	3938.7	3516.7	175835	5350	3960	150	1860	660	750	12730	163105	D

Where, T1-T16 = treatment numbers 1 up to 16. UUY = unadjusted grain yield, AGY = adjusted grain yield, NPSB = nitrogen phosphorous, sulfur and boron, ha-1 = hectare, CM = cattle manure, TVC = total varial cost, GFB GFB = gross field benefit, NB = net benefit, ETB = Ethiopian birr (one dollar = 52 ETB), MRR = marginal rate of return, ND = non dominated, D = Dominated. The market price of faba bean = 50 ETB kg-1; Cost of CAM = 1.5 ETB ha-1; Cost of NPSB fertilizer = 42.80 ETB kg-1; Labour cost for CAM application = 4 persons ha-1, each 50 ETB day-1; Labour cost for NPSB fertilizer application = 4 person ha-1, each 50 ETB day-1 (source Bonga Agricultural research center).

**Table 6:** Partial budget analysis to estimate the net benefit to combined use of CM and NPSB of Faba bean production at Boka location.

Boka												
Treatments	UUY (kg ha^−1^)	AGY (kg ha^−1^	GFB (ETB)	VC NPSB (ETB)	VC CAM (ETB)	Transportation cost (ETB)		Application cost ETB		TVC (ETB)	NFB (ETB)	MRR (%)
						NPSB (ETB)	CAM (ETB)	NPSB (ETB)	CAM (ETB)			
T 1	2720	2428.6	121430	0	0	0	0	0	0	0	121430	
T 2	3000.5	2679	133950	0	1320	0	620	0	250	2190	131760	ND
T 5	3138.6	2702.3	135115	2140	0	50	0	220	0	2410	132705	ND
T 3	3190.4	2848.6	142430	0	2640	0	1240	0	500	4380	138050	ND
T 6	3271.5	2821	141050	2140	1320	50	620	220	250	4600	136450	D
T 9	3206.1	2862.6	143130	4280	0	100	0	440	0	4820	138310	ND
T 13	3235.7	2889	144450	5350	0	150	0	660	0	6160	138290	D
T 4	3426.8	2959.6	147980	0	3960	0	1860	0	750	6570	141410	ND
T 7	3351.7	2992.6	149630	2140	2640	50	1240	220	500	6790	142840	ND
T 10	3332.7	2975.6	148780	4280	1320	100	620	440	250	7010	141770	D
T 14	3484.3	3111	155550	5350	1320	150	620	660	250	8350	147200	ND
T 8	3497.4	3122.67	156134	2140	3960	50	1860	220	750	8980	147154	D
T 11	3504	3128.6	156430	4280	2640	100	1240	440	500	9200	147230	ND
T 15	3997.3	3569	178450	5350	2640	150	1240	660	500	10540	167910	ND
T 12	3641.8	3251.6	162580	4280	3960	100	1860	440	750	11390	151190	D
T 16	3692.6	3297	164850	5350	3960	150	1860	660	750	12730	152120	D

Where, T1-T16 T1-T16 = treatment numbers 1 up to 16, UUY = unadjusted grain yield, AGY = adjusted grain yield, NPSB = nitrogen phosphorous, sulfur and boron, ha^−1^ = hectare, CM = cattle manure, TVC = total varial cost, GFB GFB = gross field benefit, NB = net benefit, ETB = Ethiopian birr (one dollar = 52 ETB), MRR = marginal rate of return, ND = non dominated, D = Dominated. Market price of faba bean = 50 ETB kg^−1^; Cost of CAM = 1.5 ETB ha^−1^; Cost of NPSB fertilizer = 42.80 ETB kg^−1^; Labour cost for CAM application = 4 persons ha^−1^, each 50 ETB day^−1^; Labour cost for NPSB fertilizer application = 4 person ha^−1^, each 50 ETB day^−1^ (source Bonga Agricultural research center).

Selective dominance analysis identified non-dominant treatments (T1, T2, T3, T7, T14, T15, and T1, T2, T5, T9, T4, T7, T14, T11, T15) at Alargeta and Boka locations, while the remaining treatments were deemed dominated. Control treatment yielded the lowest net benefit (132,280 and 121,430 ETB ha-1) in both Alargeta and Boka experimental sites (Table 5, Table 6). Despite the higher cost associated with NPSB blended fertilizer, manure emerged as an advantageous option for smallholder faba bean farmers in the area. Furthermore, manuring was noted as a means to amplify the economic benefits of P fertilizer application.

The combined application of CAM 5 t ha^−1^ with 150 kg NPSB blended fertilizer exhibited an MRR of 2595.1 % and 1545.3 %, surpassing the acceptable minimum MRR of 100 %. This implies a return of 25.951 and 15.453 ETB ha^−1^ for every 1 Birr ha^−1^ invested in faba bean production at both locations (Table 5, Table 6).

Notably, high net returns were linked to increased yields, while low net returns were tied to diminished yields. The analysis utilized partial budgeting to estimate net benefits, perform dominance analysis, and determine MRR for diverse treatments. Economically, the integrated application of 5 t ha-1 cattle manure with 150 kg ha^−1^ NPSB blended fertilizer proved the most feasible, delivering the highest profitability (187,775 and 167,010 ETB) compared to other treatments. This implies the obtained higher yields enhanced the efficiency of fertlzer and can raise farmers' income, resulting in better livelihoods and agricultural practices.

## 4 Conclusion and outlook

In conclusion, the study aimed to improve faba bean productivity in Ethiopia by investigating the impact of cattle manure (CAM) and nitrogen phosphorus sulfur and boron (NPSBP) application. Notable effects were observed on harvest index and grain yield across various CAM and blended NPSB fertilizer rates in Alargeta and Boka experimental areas. The highest harvest index (52.5 % and 49.8 %) resulted from applying 5 t ha^−1^ CAM with 150 kg ha^−1^ blended NPSB fertilizer, while the lowest values (42.8 % and 41.9 %) were recorded in control treatments. this implies specific combinations of cattle manure and NPSB fertilizer application of significantly enhanced crop productivity.

Similarly, the highest grain yield (3966.3 and 3569.0 kg ha^−1^) was achieved with CAM 5 t ha^−1^ and 150 kg ha^−1^ blended NPSB fertilization, contrasting with the lowest yields (2645.6 and 2428.6 kg ha^−1^) from control treatments. The study revealed significant impacts on faba bean phenology, growth, nodulation, yield components, and overall yield due to the interaction effects of CAM and blended NPSB fertilizer. Among the treatments, CAM 5 t ha^−1^ with 150 kg ha^−1^ blended NPSB consistently exhibited superior results. Economically, this treatment yielded the highest net benefit (187,775 and 167,010 ETB ha^−1^), exceeding the acceptable minimum marginal rate of return (MRR) of 100 %, with MRRs of 2595.1 % and 1545.3 % at Alargeta and Boka.

In summary, the integrated use of CAM 5 t ha^−1^ and 150 kg ha^−1^ NPSB blended fertilizer rates emerged as an economically feasible approach to enhance faba bean productivity in the study area. This recommendation provides valuable insights for resource-conscious farmers. Alternative strategies, such as CAM 5 t ha^−1^ with 100 kg ha^−1^ or 150 kg ha^−1^ NPSB fertilizer, are suggested for those with limitations.

The finding implies the potential of cattle manure and mineral NPSB The positive impacts to address food security challenges, economic viability, and Sustainable Agriculture in Ethiopia by significantly increasing faba bean production, a key staple crop. Future research should validate especially seasons with different genotypes. Exploring a wider range of CAM and NPSB fertilizer rates might be advantageous. More research is needed to investigate the mechanisms underlying these findings and the long-term consequences of various fertilizer techniques on faba bean output.

## CRediT authorship contribution statement

**Isreal Zewide:** Formal analysis, Data curation, Conceptualization. **Asrat Ademe:** Validation, Software, Resources.

## Ethics approval and consent to participate

Not applicable.

## Data availability

Data will be made available from the corresponding author on request.

## Funding

The authors declare that no funds, grants, or other support were received during the preparation of this manuscript.

## Declaration of competing interest

The authors declare the following financial interests/personal relationships which may be considered as potential competing interests: Isreal Zewide reports administrative support was provided by Mizan-Tepi University. Isreal Zewide reports a relationship with Mizan-Tepi University that includes: non-financial support and speaking and lecture fees. Isreal Zewide has patent pending to Mizan tepi unversity. NO If there are other authors, they declare that they have no known competing financial interests or personal relationships that could have appeared to influence the work reported in this paper.
